The article "IL-10 -1082 A>G (rs1800896) polymorphism confers susceptibility to pulmonary tuberculosis in Caucasians but not in Asians and Africans: a meta-analysis" was published in 2017. Journal: Biosci Rep.

# *IL-10* -1082 A>G (rs1800896) polymorphism confers susceptibility to pulmonary tuberculosis in Caucasians but not in Asians and Africans: a meta-analysis

**DOI:** 10.1042/BSR20170240

**Published:** 2017-10-27

**Authors:** Mohammed Y. Areeshi, Raju K. Mandal, Sajad A. Dar, Arshad Jawed, Mohd Wahid, Mohtashim Lohani, Aditya K. Panda, Bhartendu N. Mishra, Naseem Akhter, Shafiul Haque00

**Affiliations:** 1 Research and Scientific Studies Unit, College of Nursing and Allied Health Sciences, Jazan University, Jazan 45142, Saudi Arabia; 2 The University College of Medical Sciences and GTB Hospital, University of Delhi, Delhi 110095, India; 3 Centre for Life Sciences, Central University of Jharkhand, Ranchi 835205, Jharkhand, India; 4 Department of Biotechnology, Institute of Engineering and Technology, Lucknow 226021, Uttar Pradesh, India; 5 Department of Laboratory Medicine, Faculty of Applied Medical Sciences, Albaha University, Albaha 65431, Saudi Arabia

**Keywords:** Meta-analysis, IL-10, pulmonary tuberculosis, polymorphism, genetic models

## Abstract

Background: Earlier studies have shown that *interlukin-10* (*IL-10*) -1082 A>G gene polymorphism is implicated in susceptibility to pulmonary tuberculosis (PTB), but their results are inconsistent and inconclusive. In the present study, a meta-analysis was performed to analyze the potential association between *IL-10* -1082 A>G gene polymorphism and PTB susceptibility.

Methods: A quantitative synthesis was done using PubMed (Medline), EMBASE, and Google Scholar web databases search and meta-analysis was performed by calculating pooled odds ratios (ORs) and 95% confidence intervals (95% CIs) for all the genetic models.

Results: A total of 22 eligible studies comprising 4956 PTB cases and 6428 healthy controls were included in the analysis. We did not observe any increased or decreased risk of PTB in allelic contrast (G vs. A: *P*=0.985; OR = 1.001, 95% CI = 0.863–1.162), homozygous (GG vs. AA: *P*=0.889; OR = 1.029, 95% CI = 0.692–1.529), heterozygous (GA vs. AA: *P*=0.244; OR = 0.906, 95% CI = 0.767–1.070), dominant (GG + AG vs. AA: *P*=0.357; OR = 1.196, 95% CI = 0.817–1.752), and recessive (GG vs. AA + AG: *P*=0.364; OR = 0.921, 95% CI = 0.771–1.100) genetic models. Likewise, no association of *IL-10* -1082 A>G polymorphism with PTB risk was observed in Asian and African population for all the genetic models. Interestingly, the dominant model (GG + AG vs. AA: *P*=0.004; OR = 1.694, 95% CI = 1.183–2.425) demonstrated increased risk of PTB in Caucasian population.

Conclusions: This meta-analysis concludes that *IL-10* -1082 A>G gene polymorphism is not significantly associated with overall, Asian and African population. However, this polymorphism is associated with Caucasian population.

## Introduction

Tuberculosis (TB) caused by *Mycobacterium tuberculosis* (*M. tuberculosis* or *M. tb*) is mainly a disease of the lungs mostly of pulmonary type tuberculosis (PTB), which can easily be spread to others by coughing and breathing. Regardless of availability of various effective treatment strategies, which were assumed to eliminate this disease, recent epidemiological figures of the year 2016 shown that TB is once more on the upsurge [1]. Globally, there is a large burden of disease with 9.6 million new cases and 1.5 million people are reported to deaths in the year 2014 [1].

Approximately one-third of the world’s population is thought to be affected with *M. tuberculosis* but relatively large number of population remains with no clinical sign of the disease. However, remaining 5–15% of the infected individuals develop active disease later in life [2]. This suggests that besides *Mycobacteria* itself, the host genetic factors may regulate the differences in host susceptibility to TB [3]. The identification of host genes and genetic variations that are important in susceptibility and resistance to tuberculosis would lead to a better understanding of the pathogenesis of PTB and perhaps lead to new approaches of the disease treatment or prophylaxis.

Immune response to PTB is regulated by interactions between lymphocytes with antigen-presenting cells and the cytokines secreted by these cell types. Cytokines, their genes and receptors have been implicated in the protective immunity, pathophysiology and in the development of tuberculosis [4]. Manifestation of clinical PTB depends on balance between *T helper 1* (*Th1*) cytokines associated with resistance to infection and *Th2* cytokines with progressive disease [5].

*IL-10* gene maps on the long arm of chromosome 1 (1q31-1q32) locus and produced by both myeloid cells and T cells. *IL-10* signals through a receptor complex consisting of two subunits: *IL-10*R1, induced on stimulated hematopoietic cells, and the *IL-10*R2, constitutively expressed on most cells and tissues [6].

*IL-10*, an anti-inflammatory cytokine prevents the protective immune response to pathogens by blocking the production of proinflammatory cytokines, such as *TNF-α* and *Th1*-polarizing cytokine IL-*12*, by directly acting on antigen-presenting cells such as macrophages and dendritic cells [7]. *IL-10* may also inhibit phagocytosis and microbial killing by limiting the production of reactive oxygen and nitrogen intermediates in response to *IFN-γ* and *Th1* induced response to TB [8,9]. *IL-10* was shown to be elevated in the lungs and serum of PTB patients [10].

The production of cytokines can be modulated both by the stimuli present in the local environment as well as by the genetic factors. Both, *in vitro* and *in vivo* studies have demonstrated that the presence of polymorphisms within the coding or noncoding sequences of cytokine genes can alter the efficiency of transcription of these genes and thus the production of cytokines. Interindividual variations in *IL-10* production are genetically contributed by polymorphisms within the promoter region. The polymorphism -1082 A>G occurs within a putative Ets (E26 transformation-specific) transcription factor-binding site and may affect the binding of this transcriptional factor and therefore altered levels of this cytokine and may alter *Th1*/ *Th2* balance with major implications in tuberculous infection [11,12].

A number of clinical and genetic studies have been performed to consider the effect of *IL-10* -1082 A>G (rs1800896) gene polymorphism on the development of PTB [13–34]. Results published from previous studies are either conflicting or contradictory in nature and still it is unclear whether this polymorphism is associated with increased or decreased risk of PTB infection [13–34]. Inconsistency in the results across many of the studies could possibly be due to the ethnicity of the population, sample size, and individual studies that have low power to evaluate the overall effect. To overcome this situation, nowadays meta-analysis statistical tool is in use to explore the risk factors associated with the genetic diseases, because it employs a quantitative method of pooling the data collected from individual studies where sample sizes are small to provide reliable conclusions. Hence, in the present study, a meta-analysis was performed to evaluate the effect of *IL-10* -1082 A>G gene polymorphism on the risk of overall PTB development and its ethnicity-wise distribution.

## Materials and methods

### Literature search strategy

We performed a PubMed, Medline, EMBASE, and Google Scholar web databases search covering all research articles published with a combination of the following key words, i.e. *IL-10, Interleukin-10* gene (polymorphism OR mutation OR variant) AND tuberculosis susceptibility or TB or Pulmonary tuberculosis or PTB (last updated on June 2016). We examined potentially pertinent genetic association studies by examining their titles and abstracts, and procured the most relevant publication matching with the eligible criteria for a closer examination. Besides the online database search, the references given in the selected research articles were also screened for other potential articles that may have been missed in the primary search.

### Inclusion and exclusion criteria

In order to minimize heterogeneity and facilitate the proper interpretation of this study, published articles included in the current meta-analysis had to meet all the following criteria, i.e.

- they must have done case–control studies between *IL-10*-1082 A>G gene polymorphism and PTB risk,
- clearly described confirmed PTB patients and PTB free controls
- have available genotype frequency in the both cases and controls
- published in the English language
- data collection and analysis methodology should be statistically acceptable
- additionally, when the case–control study was included in more than one research article using the same subject series, we selected the research study that incorporated the largest number of individuals.

The major reasons for study exclusion were:

- duplicate or overlapping publication
- study design based on only PTB cases
- genotype frequency not reported
- data of review or abstract

### Data extraction and quality assessment

For each retrieved study, the methodological quality assessment and data extraction were independently abstracted in duplicate by two independent investigators (SAD & RKM) using a standard protocol. Data collection form was used to confirm the accuracy of the collected data by strictly following the inclusion/exclusion criteria as stated above. In case of disagreement between the above mentioned two investigators on any item related with the data collected from the selected studies, the issue was fully debated and deliberated with the investigators to attain a final consensus. Also, in case failure of reaching consensus between the two investigators, an agreement was achieved following an open discussion with the adjudicator (SH). The major characteristics abstracted from the retrieved publications included the name of first author, publication year, the country of origin, source of cases and controls, number of cases and controls, study type, genotype frequencies, and association with pulmonary TB.

### Quality assessment of the included studies

Methodological quality evaluation of the selected studies was performed independently by two investigators (RKM & SAD) by following the Newcastle–Ottawa Scale (NOS) of quality assessment [35]. The NOS quality assessment criteria included three major aspects: (i) subject selection: 0–4 points, (ii) comparability of subject: 0–2 points, and (iii) clinical outcome: 0–3 points. Selected case–control studies that gained five or more stars were considered as of moderate to good quality [36].

### Statistical analysis

In order to evaluate the association between the *IL-10* -1082 A>G gene polymorphism and risk of developing PTB, pooled ORs and their corresponding 95% CIs were estimated. Heterogeneity assumption was examined by the chi-square-based *Q*-test [37]. Heterogeneity was considered significant at *P*-value < 0.05. The data from single comparison were combined using a fixed effects model [38], when no heterogeneity was obtained. Otherwise the random-effects model was used for the pooling of the data [39]. Moreover, *I*^2^ statistics was employed to quantify interstudy variability and larger values suggested an increasing degree of heterogeneity [40]. Hardy–Weinberg equilibrium (HWE) in the controls was calculated by chi-square test. Funnel plot asymmetry was measured by Egger’s regression test, which is a type of linear regression approach to measure the funnel plot asymmetry on the natural logarithm scale of the OR. The significance of the intercept was measured by the *t*-test (*P*-value < 0.05 was considered as a representation of statistically significant publication bias).

A comparative assessment of ‘meta-analysis’ based programs was done by using weblink http://www.meta-analysis.com/pages/comparisons.html. The Comprehensive Meta-Analysis (CMA) Version 2 software program (Biostat, U.S.A.) was utilized to perform all the statistical analysis involved in this meta-analysis.

## Results

### Characteristics of the published studies

A total of 22 articles were lastly selected after literature search from the PubMed (Medline), EMBASE, and Google Scholar web databases. All retrieved articles were inspected carefully by reading their titles and abstracts, and the full-texts for the potentially relevant publications were further checked for their aptness of inclusion in this meta-analysis (Figure 1: PRISMA 2009 Flow Diagram). All the included 22 studies follow the preset eligible criteria of the study inclusion and clearly stated about sample sizes, genotypes, inclusion criteria of PTB patients, and healthy controls. All the studies included in this meta-analysis had recruited HIV free subjects.

**Figure 1:** PRISMA flow-diagram The selection process (inclusion/exclusion) of the studies dealing with *IL10* -1082 A>G (rs1800871) gene polymorphism and PTB risk.

Research articles either showing *IL-10* polymorphism to predict survival in PTB patients or considering *IL-10* variants as indicators for response to therapy were excluded straightaway. Similarly, studies investigating the levels of *IL-10* mRNA or protein expression or relevant review articles were also excluded from this meta-analysis. We included only case–control or cohort design studies stating the frequency of all three genotypes. Besides the database search, the supporting references available in the retrieved articles were also checked for other potential studies. After careful screening and following the inclusion and exclusion criteria, 22 eligible original published studies were finally considered for the present study (Table 1). Distribution of genotypes, HWE *P*-values in the controls, and susceptibility toward PTB have been shown in Table 2. All the selected studies (22 in number) were examined for the overall quality following the NOS and most of the studies (>80%) scored five stars or more, indicating a modest to good quality (Table 3).

**Table 1:** Main characteristics of all studies included in the present meta-analysis

First author and year [Ref.]	Country	Ethnicity	Controls	Cases	Study	Genotyping technique
Hu et al., 2015 [13]	China	Asian	480	120	HB	ARMS PCR
Feng et al., 2014 [14]	China	Asian	191	191	HB	PCR-RFLP
García-Elorriaga et al., 2013 [15]	Mexico	Mixed	47	40	HB	TaqMan
Akgunes et al., 2011 [16]	India	Asian	30	30	HB	PCR Probe
Liang et al., 2011 [17]	China	Asian	78	112	HB	SNaPshot assay
Ansari et al., 2011 [18]	Pakistan	Asian	166	102	HB,PB	ARMS PCR
Ben-Selma et al., 2011 [19]	Tunisia	African	95	76	HB	ARMS PCR
Taype et al., 2010 [20]	Peru	Caucasian	510	500	PB	PCR-RFLP
Mosaad et al., 2010 [21]	Egypt	African	98	26	HB	ARMS PCR
Thye et al., 2009 [22]	Ghana	African	1968	1541	HB	FRET
Ansari et al., 2009 [23]	Pakistan	Asian	188	111	HB	ARMS PCR
Trajkov et al., 2009 [24]	Macedonia	Caucasian	301	75	HB, PB	PCR-SSP
Selvaraj et al., 2008 [25]	India	Asian	183	155	HB	ARMS PCR
Wu et al., 2008 [26]	China	Asian	111	183	PB	PCR RFLP
Anand et al., 2007 [27]	India	Asian	143	132	HB	ARMS PCR
Oh et al., 2007 [28]	Korea	Asian	117	145	HB	ARMS PCR
Amirzargar et al., 2006 [29]	Iran	Asian	123	41	HB	PCR-SSP
Shin et al., 2005 [30]	Korea	Asian	871	459	HB	MAPA
Scola et al., 2003 [31]	Italy	Caucasian	114	45	HB	ARMS PCR
López-Maderuelo et al., 2003 [32]	Spain	Caucasian	100	113	HB	ARMS PCR
Delgado et al., 2002 [33]	Cambodia	Asian	106	358	HB	PCR-SSP
Bellamy et al., 1998 [34]	Gambia	African	408	401	HB	Hybridization

Abbreviations: ARMS PCR, amplification-refractory mutation system polymerase chain reaction; FRET, fluorescence resonance energy transfer; HB, hospital based; MAPA, multiplex automated primer extension analysis; PB, population based; PCR-SSP, polymerase chain reaction with a sequence specific primers.

**Table 2:** Genotypic distribution of *IL-10* -1082 A>G (rs1800896) gene polymorphism included in the meta-analysis

First author and year	Controls				Cases				
	Genotype			Minor allele	Genotype			Minor allele	HWE
	AA	GA	GG	MAF	AA	GA	GG	MAF	*P*-value
Hu et al., 2015	262	196	22	0.250	82	34	4	0.175	0.35
Feng et al., 2014	171	18	2	0.057	164	24	3	0.078	0.08
Elorriaga et al., 2013	25	18	4	0.276	27	11	2	0.187	0.01
Akgunes et al., 2011	17	13	0	0.216	15	9	6	0.350	0.26
Liang et al., 2011	69	9	0	0.057	100	12	0	0.053	0.11
Ansari et al., 2011	31	118	17	0.457	23	64	15	0.460	0.04
Ben-Selma et al., 2011	60	26	9	0.231	30	33	13	0.388	0.01
Taype et al., 2010	347	153	10	0.169	333	147	20	0.187	0.28
Mosaad et al., 2010	8	88	2	0.469	0	16	10	0.692	0.13
Thye et al., 2009	1048	783	140	0.269	794	630	117	0.280	0.27
Ansari et al., 2009	32	136	20	0.468	21	71	19	0.490	0.03
Trajkov et al., 2009	70	212	17	0.411	17	48	10	0.453	0.04
Selvaraj et al., 2008	108	69	6	0.221	102	42	5	0.174	0.83
Wu et al., 2008	104	18	0	0.073	48	12	1	0.114	0.98
Anand et al., 2007	73	61	6	0.260	74	55	3	0.231	0.01
Oh et al., 2007	45	53	19	0.388	98	43	4	0.175	0.95
Amirzargar et al., 2006	18	79	5	0.436	7	31	2	0.437	0.04
Shin et al., 2005	718	124	9	0.083	394	53	2	0.063	0.47
Scola et al., 2003	13	77	24	0.548	6	22	17	0.622	0.05
Maderuelo et al., 2003	21	50	29	0.540	33	47	33	0.501	0.91
Delgado et al., 2002	39	64	3	0.330	86	259	11	0.394	0.06
Bellamy et al., 1998	179	184	45	0.335	165	185	11	0.286	0.07

Abbreviations: HWE, Hardy–Weinberg equilibrium; MAF, minor allele frequency;.

**Table 3:** Quality assessment conducted according to the NOS for all the studies included in the meta-analysis

First author and year [Ref.]	Quality indicators		
	Selection	Comparability	Exposure
Hu et al., 2015 [13]	***	*	**
Feng et al., 2014 [14]	***	*	**
García-Elorriaga et al., 2013 [15]	***	*	**
Akgunes et al., 2011 [16]	**	*	**
Liang et al., 2011 [17]	****	**	**
Ansari et al., 2011 [18]	***	*	**
Ben-Selma et al., 2011 [19]	****	*	**
Taype et al., 2010 [20]	****	*	**
Mosaad et al., 2010 [21]	***	*	**
Thye et al., 2009 [22]	****	**	**
Ansari et al., 2009 [23]	***	*	**
Trajkov et al., 2009 [24]	***	*	**
Selvaraj et al., 2008 [25]	****	*	**
Wu et al., 2008 [26]	***	*	***
Prabhu Anand et al., 2007 [27]	***	*	***
Oh et al., 2007 [28]	**	*	**
Amirzargar et al., 2006 [29]	**	*	**
Shin et al., 2005 [30]	****	*	**
Scola et al., 2003 [31]	**	*	**
López-Maderuelo et al., 2003 [32]	***	*	**
Delgado et al., 2002 [33]	***	**	**
Bellamy et al., 1998 [34]	***	*	**

### Publication bias

Begg’s funnel plot and Egger’s test were performed to examine the publication bias among the selected studies for the present meta-analysis. The funnel plots were almost symmetric for both the Begg’s test and Egger’s test (Figure 2). The findings showed lack of publication bias among all comparison models (Table 4).

**Figure 2:** Funnel plot: Begg’s Funnel plot for overall analysis.

**Table 4:** Statistics to test publication bias and heterogeneity in meta-analysis: overall analysis

Comparisons	Egger’s regression analysis			Heterogeneity analysis			Model used for the meta-analysis
	Intercept	95% confidence interval	*P*-value	*Q*-value	*P*_heterogeneity_	*I*^2^ (%)	
G vs. A	0.134	−1.53 to 1.80	0.868	78.171	0.001	73.13	Random
GG vs. AA	0.261	−1.12 to 1.64	0.696	60.855	0.001	67.135	Random
AG vs. AA	−0.494	−1.68 to 0.69	0.396	48.356	0.001	56.572	Random
GG + AG vs. AA	−0.293	−1.63 to 1.04	0.651	60.090	0.001	65.052	Random
GG vs. AA + AG	0.420	−1.10 to 1.94	0.570	69.612	0.001	71.270	Random

### Test of heterogeneity

In order to test heterogeneity among the selected studies, *Q*-test and *I*^2^ statistics were employed. Significant heterogeneity was detected in all models. Therefore, random effects model was applied to synthesize the data (Table 4).

### Sensitivity analysis

Sensitivity analysis was performed to assess the influence of each individual study on the pooled OR by deleting one single study each time. The results showed that no individual affected the pooled OR significantly, suggesting stability of this meta-analysis (Figure 3).

**Figure 3:** Forest Plot: Sensitivity analysis for overall analysis.

### Quantitative synthesis

We pooled all the 22 studies together which resulted into 4956 confirmed PTB cases and 6428 controls, for the assessment of overall association between the *IL-10* -1082 gene polymorphism and risk of developing PTB. The pooled ORs from the overall studies indicated no association with increased or decreased risk between *IL-10* -1082 A>G gene polymorphism and PTB susceptibility in allelic contrast (G vs. A: *P*=0.985; OR = 1.001, 95% CI = 0.863–1.162), homozygous (GG vs. AA: *P*=0.889; OR = 1.029, 95% CI = 0.692–1.529), heterozygous (GA vs. AA: *P*=0.244; OR = 0.906, 95% CI = 0.767–1.070), dominant (GG + AG vs. AA: *P*=0.357; OR = 1.196, 95% CI = 0.817–1.752), and recessive (GG vs. AA + AG: *P*=0.364; OR = 0.921, 95% CI = 0.771–1.100) genetic models, respectively (Figures 3 and 4).

**Figure 4:** Forest plot: Overall analysis showing OR with 95% CI to evaluate the association of the *IL10* -1082 A>G (rs1800871) gene polymorphism and PTB risk. Black squares represent the value of OR and the size of the square indicates the inverse proportion relative to its variance. Horizontal line is the 95% CI of OR.

### Subgroup analysis

We have performed subgroup analysis based on ethnicity to explore the effect of ethnicity (Asian, African, and Caucasian) in the risk between *IL-10* -1082 A>G and PTB risk.

### Asian population

In Asian population, 13 studies were included and heterogeneity was observed in all the genetic models (Table 5). We performed analyses using random effect models for all the genetic models and no significant association of PTB susceptibility in all genetic models was detected in allele model (G vs. A: *P*=0.466; OR = 0.917, 95% CI = 0.726–1.158), homozygous model (GG vs. AA: *P*=0.602; OR = 0.853, 95% CI = 0.4710–1.547), heterozygous model (GA vs. AA: *P*=0.170; OR = 0.839, 95% CI = 0.652–1.078), dominant model (GG + AG vs. AA: GG vs. AA + AG: *P*=0.836; OR = 0.945, 95% CI = 0.554–1.613), and recessive model (GG vs. AA + AG: *P*=0.282; OR = 0.858, 95% CI = 0.650– 1.134) (Figure 5).

**Figure 5:** Forest plot: Data from the Asian population showing OR with 95% CI to evaluate the association of the *IL10* -1082 A>G (rs1800871) gene polymorphism and PTB risk. Black squares represent the value of OR and the size of the square indicates the inverse proportion relative to its variance. Horizontal line is the 95% CI of OR.

**Table 5:** Statistics to test publication bias and heterogeneity in the present meta-analysis: Asian population

Comparisons	Egger’s regression analysis			Heterogeneity analysis			Model used for the meta-analysis
	Intercept	95% confidence interval	*P*-value	*Q*-value	*P*_heterogeneity_	*I*^2^ (%)	
G vs. A	1.686	−2.38 to 5.75	0.380	44.674	0.001	73.139	Random
GG vs. AA	1.018	−1.08 to 3.88	0.446	24.674	0.010	55.419	Random
AG vs. AA	0.883	−2.29 to 4.06	0.552	28.851	0.004	58.409	Random
GG+AG vs. AA	1.672	−1.85 to 5.19	0.318	37.372	0.001	67.890	Random
GG vs. AA+AG	0.025	−2.42 to 2.47	0.981	22.603	0.020	51.334	Random

### African population

In African population four studies were found. Publication bias was not significant but heterogeneity was found significant and conducted analyses using random effect models for all the genetic models (Table 6). We found no association with PTB risk in allele model (G vs. A: *P*=0.165; OR = 1.300, 95% CI = 0.898–1.883), homozygous model (GG vs. AA: *P*=0.569; OR = 1.407, 95% CI = 0.434–4.562), heterozygous model (GA vs. AA: *P*=0.128; OR = 1.101, 95% CI = 0.973–1.246), dominant model (GG + AG vs. AA: *P*=0.438; OR = 1.614, 95% CI = 0.482–5.412), and recessive model (GG vs. AA + AG: *P*=0.244; OR = 1.240, 95% CI = 0.863–1.783) genetic models (Figure 6).

**Figure 6:** Forest plot: Data from the African population showing OR with 95% CI to evaluate the association of the *IL10* -1082 A>G (rs1800871) gene polymorphism and PTB risk. Black squares represent the value of OR and the size of the square indicates the inverse proportion relative to its variance. Horizontal line is the 95% CI of OR.

**Table 6:** Statistics to test publication bias and heterogeneity in the present meta-analysis: African population

Comparisons	Egger’s regression analysis			Heterogeneity analysis			Model used for the present meta-analysis
	Intercept	95% confidence interval	*P*-value	*Q*-value	*P*_heterogeneity_	*I*^2^ (%)	
G vs. A	2.415	−7.48 to 12.31	0.403	21.824	0.001	86.254	Random
GG vs. AA	1.047	−11.12 to 13.21	0.746	26.345	0.001	88.613	Random
AG vs. AA	1.562	−2.28 to 5.40	0.222	6.646	0.084	54.862	Fixed
GG + AG vs. AA	1.610	−4.12 to 7.34	0.350	10.073	0.018	70.216	Random
GG vs. AA + AG	1.486	−13.42 to 16.40	0.709	35.484	0.001	91.545	Random

### Caucasian population

In Caucasian population four studies were included. Publication bias and heterogeneity were not significant, hence fixed effect models were applied for all the genetic models (Table 7). We potentially found association of PTB risk with dominant model (GG + AG vs. AA: *P*=0.004; OR = 1.694, 95% CI = 1.183– 2.425). Whereas, other genetic models, i.e. allele (G vs. A: *P*=0.236; OR = 1.103, 95% CI = 0.938–1.298), homozygous model (GG vs. AA: *P*=0.098; OR = 1.439, 95% CI = 0.935–2.215), heterozygous model (GA vs. AA: *P*=0.446; OR = 0.915, 95% CI = 0.729–1.150), and recessive model (GG vs. AA + AG: *P*=0.926; OR = 0.990, 95% CI = 0.794–1.233) did not show any increased or decreased risk of PTB with *IL-10* -1082 A>G gene polymorphism (Figure 7).

**Figure 7:** Forest plot: Data from the Caucasian population showing OR with 95% CI to evaluate the association of the *IL10* -1082 A>G (rs1800871) gene polymorphism and PTB risk. Black squares represent the value of OR and the size of the square indicates the inverse proportion relative to its variance. Horizontal line is the 95% CI of OR.

**Table 7:** Statistics to test publication bias and heterogeneity in the present meta-analysis: Caucasian population

Comparisons	Egger’s regression analysis			Heterogeneity analysis			Model used for the present meta-analysis
	Intercept	95% confidence interval	*P*-value	*Q*-value	*P*_heterogeneity_	*I*^2^ (%)	
G vs. A	0.158	−8.42 to 8.74	0.940	2.616	0.455	0.001	Fixed
GG vs. AA	2.859	−16.58 to 22.30	0.590	5.366	0.147	44.089	Fixed
AG vs. AA	−1.361	−4.15 to 1.42	0.170	2.446	0.485	00.001	Fixed
GG + AG vs. AA	−1.031	−4.68 to 2.62	0.348	2.235	2.235	0.5250	Fixed
GG vs. AA + AG	8.205	3.75 to 12.65	0.015	4.744	0.192	36.760	Fixed

## Discussion

Although various mechanisms have been described for the development of a protective immune response that restricts and controls the infection and thus prevents the progression of the active disease, the reasons underlying active disease progression remain poorly understood [41]. Candidate gene approach and association studies have identified various host genetic factors that affect the susceptibility to TB [41]. As an immune response modulator, IL-10 has a crucial role to suppress proinflammatory cytokine responses by the innate and adaptive immune systems [42]. *IL-10* is also thought to play an important regulatory role in many bacterial infections [43,44]. Immunoregulatory genes are very important in modulating the host susceptibility to PTB because the first line of defense against *M. tuberculosis* involves the identification and uptake of the bacterium by macrophages and dendritic cells [45].

As we know that PTB is one of the most common infectious diseases with a high morbidity and mortality [1]. A well-established genetic marker surely would have a significant influence in screening and prevention of PTB. Cytokine polymorphism has been considered to be of important roles in host genetic factors. Among them, *IL-10* is an essential pleiotropic cytokine which takes part in immunoregulatory activities. Lately, *IL-10* gene has been widely studied and some studies suggested that the *IL-10* -1082 A>G polymorphism is associated with PTB susceptibility, but the results are inconsistent. The results of studies generated could be having insufficient statistical power of individual studies with small sample sizes or variations that existed in different population. Therefore, we conducted this meta-analysis to provide more accurate statistical evidence of association between *IL-10* -1082 A>G polymorphism and PTB susceptibility. Pooled ORs generated from large sample size and sufficient statistical power from various studies have the advantage of reducing random errors [46].

In the present study, we have included 22 studies with all the preset eligible criteria of sample size, genotype, inclusion criteria of PTB patients, and healthy controls. Most of the included studies scored five or more stars in NOS quality score assessment and suggested good to moderate quality by clearly stating about the sample size, genotype, inclusion criteria of PTB patients, and healthy controls.

Overall, we found that there was no association between *IL-10* -1082 A>G polymorphism and PTB susceptibility under any genetic models in overall analysis.

These observations suggested that the *IL-10* -1082 A allele leads to increased resistance to PTB. Studies carried out on mice observed that overexpression of *IL-10* may not be important for susceptibility to initial infection with *M. tb* but may play a role in reactivation of the latent disease [47]. Other studies also reported no association between the said polymorphism and resistance to TB [48,49].

During the subgroup analysis, we found that *IL-10* -1082 A>G polymorphism has no role of increasing or decreasing PTB susceptibility in Asian and African populations. Interestingly, significant association was found with dominant model. This result implied that among different ethnicities, the same gene polymorphism may act differently in PTB susceptibility. Tuberculosis report clarified racial differences of susceptibility to TB [50]. Thus, the current results of the present study might attribute the racial differences and reflect the existence of racial differences of TB.

However, the susceptibility toward PTB is polygenic and multiple candidate genes are likely to be involved in determining resistance or susceptibility to TB [51]. Due to multifactorial nature of TB infection and complex nature of the immune system, *IL-10* -1082 A>G genetic polymorphism cannot be solely responsible for the predisposition of PTB.

In the present study, significant heterogeneity was found between the selected studies in the test of heterogeneity. This discordance may be related to the ethnic origin of the patients as ethnicity-specific genetic variations may influence the host immunity to PTB. Nevertheless, some limitations also need to be addressed. First, we only included studies published in the English language, abstracted and indexed by the selected electronic databases were included for data analysis; it is possible that some pertinent studies published in other languages and indexed in other electronic databases may have missed. Second, the abstracted data were not stratified by other factors, e.g. HIV status or severity of the TB infection, and our results were based on unadjusted parameters. Third, we did not test for gene–environment interactions because of inadequate data available in the published reports. Despite above limitations, there are some advantages of the present study. First, the present meta-analysis was comprised with more number of studies which increased the statistical power of the study and ultimately reached at robust conclusion. Second, no publication bias was observed and further sensitivity analysis also supported our results more reliably.

Also, all the included studies were of good to modest quality fulfilling the preset needful criteria as tested by NOS quality score evaluation scale.

## Conclusions

In conclusion, this meta-analysis demonstrated that *IL-10* -1082 A>G gene polymorphism is not associated with PTB risk in overall, Asian and African population. Our result provided evidence that G allele carrier is associated with PTB in Caucasian population. In the near future, because of significant public health impact of PTB, larger studies are warranted to identify the host genes with their functional allele controlling the response to mycobacterial infections. This will help in the identification of the host genetic factors for the susceptibility to PTB, and would greatly help in the global control of this infectious disease.

## Abbreviations

CI: confidence interval
HWE: Hardy–Weinberg equilibrium
IFN-y: Interferon gamma
IL-10: interlukin-10
NOS: Newcastle–Ottawa Scale
OR: odds ratio
PTB: pulmonary tuberculosis
Th1: T helper 1
TNF-a: Tumor necrosis factor - alpha
